# A Simple and Portable Personal Glucose Meter Method Combined with Molecular Docking for Screening of Lipase Inhibitors

**DOI:** 10.1155/2022/4430050

**Published:** 2022-09-22

**Authors:** Hao Zhang, Feng-Qing Yang, Jian-Li Gao

**Affiliations:** ^1^Chongqing Key Laboratory of High Active Traditional Chinese Drug Delivery System, Chongqing Medical and Pharmaceutical College, Chongqing 401331, China; ^2^School of Chemistry and Chemical Engineering, Chongqing University, Chongqing 401331, China; ^3^Zhejiang Chinese Medical University, Hangzhou 310053, Zhejiang, China

## Abstract

With the increase of obesity incidence, the development of antiobesity drugs has aroused extensive interest. In this study, a simple and portable personal glucose meter (PGM) method based on the lipase-mediated reaction combined with molecular docking was developed for the screening of lipase inhibitors. Lipase can catalyse the hydrolysis of 4-acetamidophenyl acetate to form acetaminophen, which can directly trigger the reduction of K_3_[Fe(CN)_6_] to K_4_[Fe(CN)_6_] in the glucose test strips and generate an electrical signal that can be detected by the PGM. When lipase inhibitors exist, the yield of acetaminophen will be reduced and results in a corresponding decrease of the PGM signal. Therefore, the activity of lipase can be measured by the PGM. After optimization of the experimental conditions, the inhibitory activity of fourteen small-molecule compounds and fifteen natural product extracts on lipase were evaluated by the developed PGM method. The results indicate that tannic acid, (-)-epigallocatechin gallate, (-)-epigallocatechin, (-)-epicatechin gallate, and epicatechin have good inhibitory effect on lipase (% of inhibition higher than 40.0%). Besides, the natural product extracts of Galla Chinensis, lemon, and Rhei Radix et Rhizoma have a good inhibitory effect on lipase with % of inhibition of (97.5 ± 0.6)%, (88.1 ± 0.7)%, and (79.1 ± 1.6)%, respectively. Finally, the binding sites and modes of six small-molecule compounds on lipase were investigated by the molecular docking study. The results show that the developed PGM method is an effective approach for the discovery of potential lipase inhibitors.

## 1. Introduction

Obesity is classified as an epidemic by the World Health Organization that affects many people [1]. It was estimated that about 10,000 deaths of American adults are related to the obesity each year [2]. In addition, obesity may lead to a series of complications such as hypertension, diabetes [3–6], and kidney disease [7], which seriously endanger human health. Usually, obesity is caused by excessive accumulation of fat [8]. Triglycerides is one of the most abundant types of fat in the human body and an important part of dietary fat. Therefore, inhibiting the digestion of triglycerides to reduce the fat absorption can be considered as a promising weight loss method [9]. Lipase is an esterase that can hydrolyse more than half of dietary fat to free fatty acids or monoglycerides [10, 11], and the weight loss may be achieved through inhibiting its activity [12]. However, the currently recognized antiobesity drugs are often accompanied by serious damage to the human body, such as diarrhoea and other gastrointestinal side effects [13]. In recent years, natural product extracts have received much attention due to their rich in biological activities [14]. Previous studies show that mulberry leaf [15], *Polygonum cuspidatum* [16], and other natural product extracts have a good inhibitory activity on lipase. Therefore, it is of great significance to discover more safe and effective lipase inhibitors from natural products. To date, a variety of screening methods for lipase inhibitors have been established based on high-performance liquid chromatography-mass spectrometry [17–19] and capillary electrophoresis [20]. However, these methods are usually complicated and expensive, require professional operators, and their results may be interfered by the background signal of the sample.

The point-of-care testing (POCT) technology is a popular analytical method that can obtain accurate and effective results [21]. As one of the most successful and effective tools of POCT, personal glucose meter (PGM) is widely used for its less analysis time, simple operation, portability, and low cost [22]. Moreover, many methods based on the PGM for measuring analytes other than glucose have been reported, including DNA [23], enzyme activity and their inhibitors [24–26], and heavy metals [27]. For example, a green PGM method was developed for direct determination of hydrogen peroxide and hypochlorite by us [28]. In the method, acetylcholinesterase catalyses the hydrolysis of acetylthiocholine iodide (ATCI) to generate thiocholine iodide, which triggers the reduction of K_3_[Fe(CN)_6_] to K_4_[Fe(CN)_6_] in the glucose test strips and generates a PGM detectable signal. The PGM readout is reduced after the hydrogen peroxide or hypochlorite being preincubated with the ATCI. The limit of quantitation are 1.7 mM and 0.9 mM for hydrogen peroxide and hypochlorite, respectively.

In this study, a fast and simple PGM method was developed for the screening of lipase inhibitors, which is based on the lipase-catalysing hydrolysis of 4-acetamidophenyl acetate to form acetaminophen. The acetaminophen can directly trigger the reduction of K_3_[Fe(CN)_6_] to K_4_[Fe(CN)_6_] and generate a PGM detectable signal. After the addition of lipase inhibitors, the yield of the hydrolysing product (acetaminophen) decreases and results in a decrease of the PGM readout. The experimental conditions, including the relationship between PGM readout and 4-acetamidophenyl acetate concentration, incubation time, temperature, and lipase concentration were systematically optimized. Then, the inhibitory activity of fourteen small-molecule compounds and fifteen natural product extracts on lipase were evaluated by the developed method, and the binding mode and position of six small-molecule compounds on lipase were further investigated by the molecular docking study. The proposed PGM-based method can be used for the inhibitor screening without any modification of lipase and substrate, as well as the complicated experimental operation.

## 2. Materials and Methods

### 2.1. Chemicals and Materials

Lipase from *Candida rugosa* (enzyme activity ≥700 U/mg) and *α*-arbutin were purchased from Shanghai Macklin Co., Ltd. (Shanghai, China). 4-Acetamidophenyl acetate was purchased from Bide Pharmatech Ltd. (Shanghai, China). (−)-Epigallocatechin gallate (EGCG), (−)-epigallocatechin (EGC), (−)-epicatechin gallate (ECG), and epicatechin (EC) were purchased from Chengdu Must Bio-Technology Co., Ltd. (Chengdu, China). Rosmarinic acid, puerarin 6″-O-xyloside, syringin, and coumarin were purchased from Chengdu Purechem Standard Co., Ltd. (Chengdu, China). (−)-Catechin hydrate and 2,3,5,4′-tetrahydroxy stilbene-2-Ο-*β*-D-glucoside (TSG) were purchased from Shanghai Yuanye Biological Technology Co., Ltd. (Shanghai. China). Tannic acid, caffeic acid, and trans-4-hydroxycinnamic acid were purchased from Shanghai Aladdin Biochemical Technology Co., Ltd. (Shanghai, China). Trans-Cinnamaldehyde was purchased from Shanghai Meryer Chemical Technology Co., Ltd. (Shanghai, China). Ethanol absolute was purchased from Chongqing Chuandong Chemical Co., Ltd. (Chongqing, China). Lemon piece was purchased from Sichuan Living Pharmaceutical Co., Ltd. Besides, fourteen natural product pieces were purchased from Kangmei Pharmaceutical Co., Ltd. (Guangdong, China).

### 2.2. Instrumentation

The PGM of Sannuo+ and glucose test strips (Glucose detection range: 1.1–33.3 mM) were purchased from Sinocare Inc. (Hunan, China). The drying oven (DHG-9035A) was purchased from Shanghai Yiheng Scientific Instrumental Co., Ltd. (Shanghai, China). The ultrasonic cleaner (UC–2H) was purchased from Shanghai Titan Scientific Co., Ltd. (Shanghai, China). RHP-100 high-speed multifunctional crusher was purchased from Yongkang Ronghao Industry and Trade Co., Ltd. (Zhejiang, China).

### 2.3. Preparation of Solutions and Samples

Lipase solution (9.0 mg/mL) was prepared by dissolving it in deionized water. 4-acetamidophenyl acetate solution (75.0 mM) was prepared by dissolving it in alcohol-water (v/v, 1 : 1) solution. Small-molecule compound solutions were prepared by dissolving them in 1.0 mL deionized water to the final concentration of 2.0 mM. Natural product extracts were prepared by boiling water extraction. In brief, a 2.0 g of the dried natural product sample power was added into the test tube containing 10.0 mL of boiling (100°C) deionized water, and then ultrasonic extraction for 30.0 min. After that, the supernatant was collected and filtered using a 0.22-*µ*m nylon membrane filter (Shanghai Titan Scientific Co., Ltd., Shanghai, China). The extracts were deposited at a 4°C refrigerator before use.

### 2.4. Analytical Procedure for Lipase Inhibitory Activity Evaluation

For the lipase inhibitory test, 1.0 *µ*L of lipase (9.0 mg/mL) was preincubated with various kinds of inhibitors for 5.0 min. Then, 1.0 *µ*L of 4-acetamidophenyl acetate (75.0 mM) was added to initiate the enzymatic reaction and incubated at 50°C for 15.0 min. Finally, the mixture solution was measured by the PGM. On the other hand, the solution without 4-acetamidophenyl acetate was served as the control group and measured by the PGM. In brief, 1.0 *µ*L of small-molecule compounds (6.0 mM) or natural product extracts (0.2 g/mL) were mixed with 1.0 *µ*L of lipase (9.0 mg/mL) and 1.0 *µ*L of alcohol-water (v/v, 1 : 1). After incubation at 50°C for 15.0 min, the mixture solution was measured by the PGM.

### 2.5. Inhibition Kinetics Study and Method Validation

Due to the water insolubility of orlistat, EGCG was used as a model compound to investigate the inhibition kinetics of lipase. IC_50_ was determined by using different concentrations of EGCG (1.5–12.0 mM) with a constant concentration of 4-acetamidophenyl acetate. The % of inhibition *I*(%) can be calculated through the following equation.

(1) $$\begin{array}{c} I\left(\%\right)=\left(1-\frac{I_{t}-I_{b}}{I_{0}}\right)\times 100\%, \end{array}$$

where *I*_*t*_ and *I*_*o*_ represent the PGM readout in the presence and absence of inhibitor, respectively. *I*_*b*_ represents the PGM readout of the control group. The inhibition plot was established by dose-response nonlinear regression equation using Graphpad Prism 7.

*Z′* factor was used to evaluate the performance of the developed activity evaluation method, which was calculated by

(2) $$\begin{array}{c} Z^{\prime }=1-\frac{3\sigma_{s}+3\sigma_{c}}{|\mu_{s}-\mu_{c}|}, \end{array}$$

where *µ*_*s*_ and *µ*_*c*_ represent the average of the signals of standard (*s*) (no inhibition) and the negative (*c*) control (100% inhibition by the reference inhibitor), respectively. The *σ*_*s*_ and *σ*_*c*_ express the standard deviations of the data, and 100% inhibition implies that *µ*_*c*_ = 0. Accordingly, equation (2) can be simplified to equation (3). It is worth noting that the developed method is precise and reliable if the value of the *Z′* factor is higher than 0.5.

(3) $$\begin{array}{c} Z^{\prime }=1-\frac{3\sigma_{s}}{\mu_{s}}. \end{array}$$

### 2.6. Molecular Docking

The molecular docking study was used to investigate the binding sites and modes of small-molecule compounds to lipase. The known crystal lipase (PDB ID : 3ICW) was downloaded from Protein Data Bank (https://www.rcsb.org./pdb). The chemical structures were drawn and energy minimized by the Chem Office 3D. The grid box centre value was set to 40, 170, and 30 along with *X*, Y, and *Z*-axis with 0.375 Å grid spacing, and size values were set as *X* = 100, *Y* = 100, and *Z* = 100. The lowest energy of the docking complex was analysed by Discovery Studio.

## 3. Results and Discussion

### 3.1. Principle of the PGM Method Based on the Lipase-Mediated Reaction

The principle of evaluation of lipase inhibitory activity by the PGM-based method is shown in Figure 1. Lipase catalyses the hydrolysis of 4-acetamidophenyl acetate to form acetaminophen. Then, acetaminophen triggers the reduction of K_3_[Fe(CN)_6_] to K_4_[Fe(CN)_6_] and generates an electrical signal that can be detected by the PGM. When a lipase inhibitor was added, the yield of the product (acetaminophen) decreased and resulted in a remarkable decrease in the PGM readout. As shown in Figure 2, the yellow colour of K_3_[Fe(CN)_6_] became colourless after the addition of the enzymatic reaction mixture solution of lipase and 4-acetamidophenyl acetate. These results show that K_3_[Fe(CN)_6_] can be reduced to K_4_[Fe(CN)_6_] by the product of the enzymatic reaction (acetaminophen).

### 3.2. Optimization of Experimental Conditions

To obtain the optimal conditions for the enzymatic reaction, various experimental parameters, including the linear relationship between the PGM readout and 4-acetamidophenyl acetate concentration (8.0–32.0 mM), incubation time (10.0–20.0 min), the enzymatic reaction temperature (30–70°C), and lipase concentration (0.2–5.0 mg/mL), were investigated.

The relationship between the PGM readout and 4-acetamidophenyl acetate concentration is shown in Figure 3(a), the PGM readout is increased with the increase in 4-acetamidophenyl acetate concentration (12.0–32.0 mM), which exhibits an excellent linear relationship in the range of 12.0–32.0 mM. The regression equation of the PGM readout = 0.331 × C_4-acetamidophenyl acetate_  + 3.708 (*R*^2^ = 0.9971). Therefore, it is feasible to detect the product of enzymatic reaction by the PGM-based method, and the concentration between 12.0 and 32.0 mM of 4-acetamidophenyl acetate was used for further study.

As shown in Figure 3(b), the enzymatic reaction can generate enough products for a suitable PGM readout with the concentrations of 4-acetamidophenyl acetate in the range of 15.0–25.0 mM. The PGM readout has a maximum value when the final concentration of 4-acetamidophenyl acetate is 25.0 mM. On the other hand, the PGM readout of 25.0 mM 4-acetamidophenyl acetate tends to be stable after incubation for 15.0 min. Therefore, the incubation time of 15.0 min and the final 4-acetamidophenyl acetate concentration of 25.0 mM were selected for the next study.

Figure 4(a) shows that the PGM readout increases with the increase in enzymatic reaction temperature, but the PGM readout is rapidly decreased at 70°C, which may be attributed to the effect of high temperature on the enzyme activity. Moreover, the PGM readout is similar when the enzymatic reaction temperature is at 50°C and 60°C. The optimal temperature is similar to that of free lipase reported in the literature (60°C) [19]. Considering that the enzyme activity is affected by high temperature, 50°C was finally selected for further study. As shown in Figure 4(b), the PGM readout increases with the increase in lipase concentration and becomes constant after the final lipase concentration reaching 3.0 mg/mL, which was selected as the optimal concentration.

### 3.3. Screening of Lipase Inhibitors by the PGM Method

The repeatability of the method was analysed based on the relative standard deviation of the PGM readout. All measurements were performed in three replicates under the optimized conditions: the final lipase concentration of 3.0 mg/mL, final 4-acetamidophenyl acetate concentration of 25.0 mM, and incubation for 15.0 min at 50.0°C. The run-to-run repeatability of a batch (*n* = 5) of glucose strips is calculated to be 5.5%, and the repeatability using different batches of glucose strips is 5.2%. Furthermore, according to equation (3), the *Z′* factor is calculated to be 0.89 (*n* = 8). These results show that the proposed activity evaluation method is reliable and accurate.

The inhibition plot of EGCG on lipase is shown in Figure 5. The IC_50_ value is calculated to be 2.1 mM. Besides, the inhibitory activities of fourteen small-molecule compounds with the final concentration of 2.0 mM on lipase were evaluated and their % of inhibition are shown in Table 1. The results show that tannic acid, EGCG, ECG, EGC, and EC have a good inhibitory effect on lipase with the % of inhibition above 40%. Furthermore, the inhibitory activities of fifteen natural product extracts on lipase were evaluated at the concentration of 0.2 g/mL (Table 2). The results show that Galla Chinensis, lemon, and Rhei Radix et Rhizoma have a good inhibitory effect on lipase with the % of inhibition of (97.5 ± 0.6)%, (88.0 ± 0.7)% and (79.1 ± 1.6)%, respectively. In reality, the protocatechuic acid, chlorogenic acid, protocatechualdehyde, rutin, isoquercitrin, astragalin, and dicaffeoylquinic acid B in a mulberry leaf [29]; the eriocitrin, citric acid, and flavones in lemon [30]; the main components polyphenols in Galla Chinensis [31]; as well as the emodin, polydatin, quercetin, and ursolic acid in Zheng et al. [32], have been reported to possess the lipase inhibitory activity. These results not only provide insights for developing an effective way in lipase inhibitor screening, but also provide an opportunity to explore novel antiobesity drugs from natural products. However, further studies should be performed to analyse and identify the main active components of natural products with an excellent lipase inhibitory activity.

### 3.4. Molecular Docking

The molecular docking study was used to investigate the binding sites and modes of small-molecule compounds on lipase. It should be mentioned that the molecular docking study was not performed for tannic acid, which cannot be analysed by the Discovery Studio. The best-docked 3D and 2D conformations of small-molecule compounds on lipase are shown in Figure 6, and the binding energy, hydrogen bonds, and amino acid residues are gathered in Table 3. Hydrogen bonds are existed between the (−)-epigallocatechin gallate and SER128, LYS132, ASN131, and LEU93; the (−)-epigallocatechin and SER128, LYS132, LYS66, and LEU275; the (−)-epicatechin gallate and SER128, LYS132, ASN131, and LYS66; the epicatechin and SER128, PRO67, and ASP160; the rosmarinic acid and ARG272 and LYS132; as well as (+)-catechin and LEU275, LEU93, and ASP160. These results indicate that hydrogen bonds play an important role in the interactions between small-molecule compounds and lipase. Furthermore, as shown in Figure 6, it can be concluded that the hydrophobic, electrostatic, and hydrogen bonds are the main interactions between four small-molecule compounds and lipase. In addition, the binding energy of the six small-molecule compounds with lipase are all below −6.0 kcal/mol, which can explain their inhibitory effects on lipase [33].

## 4. Conclusions

A rapid and convenient method for lipase inhibitor screening using a PGM combined with molecular docking was established. Compared with other methods, the main advantage of the method for lipase inhibitor screening based on PGM is that it does not require complex operations and expensive equipment. The lipase activity analysis and inhibitory activity evaluation of small-molecule compounds or natural product extracts are as simple as measuring the glucose in blood. However, this method also has some shortcomings. First, the limited detection range of PGM (1.1–33.3 mM) may result in a narrow linear range. Second, the developed method is limited for evaluating the enzyme inhibitory activity of water-insoluble components. Fourteen small-molecule compounds and fifteen natural product extracts were investigated for their inhibitory activity on lipase. Galla Chinensis, lemon, and Rhei Radix et Rhizoma have a good inhibitory activity. In addition, the results of the molecular docking study show that hydrophobic, electrostatic, and hydrogen bonds are the main interactions between small-molecule compounds and lipase.

## Figures and Tables

**Figure 1:** Schematic illustration of the principle of the PGM method based on the lipase-mediated reaction.

**Figure 2:** The colour change of the different solutions. (a) Lipase + 4-acetamidophenyl acetate solution; (b) K_3_[Fe(CN)_6_] solution; and (c) K_3_[Fe(CN)_6_]+ lipase + 4-acetamidophenyl acetate solution.

**Figure 3:** The linear relationship between the concentration of 4-acetamidophenyl acetate and PGM readout. (a) Effects of incubation time and the concentration of 4-acetamidophenyl acetate on the PGM readout. (b) The error bars represent the standard deviations of three independent measurements.

**Figure 4:** The effect of incubation temperature (a) and the concentration of lipase (b) on the PGM readout. The error bars represent the standard deviations of three independent measurements.

**Figure 5:** The inhibition plot of EGCG on lipase. The error bars represent the standard deviations of three independent measurements.

**Figure 6:** Three-dimensional (3D) and two-dimensional (2D) binding and interaction patterns of lipase with EGCG (a), EGC (b), ECG (c), and EC (d).

**Table 1:** Inhibitory activity of fourteen small-molecule compounds on lipase determined by the developed PGM method (*n* = 3).

Compounds	Inhibition (%)	Compounds	Inhibition (%)
(−)-Epigallocatechin gallate	45.3 ± 2.2	2,3,5,4′-tetrahydroxy stilbene-2-Ο-*β*-D-glucoside	19.4 ± 3.6
Tannic acid	59.8 ± 0.8	Caffeic acid	14.9 ± 3.6
(−)-Epigallocatechin	47.2 ± 1.6	Puerarin 6″-*O*-xyloside	13.8 ± 1.8
(−)-Epicatechin gallate	46.5 ± 2.2	Coumarin	12.8 ± 1.8
Epicatechin	42.8 ± 1.8	trans-4-hydroxycinnamic acid	5.4 ± 1.3
Rosmarinic acid	39.3 ± 3.0	*α*-arbutin	3.1 ± 1.6
(+)-catechin	32.7 ± 1.6	trans-cinnamaldehyde	1.7 ± 3.0

**Table 2:** Inhibitory activity of fifteen natural product extracts on lipase determined by the developed PGM-based method (*n* = 3).

Extracts	Inhibition (%)	Extracts	Inhibition (%)
Galla chinensis	97.5 ± 0.6	Paeoniae radix alba	36.5 ± 1.2
Lemon	88.1 ± 0.7	Arnebiae radix	36.3 ± 2.3
Rhei radix et rhizoma	79.1 ± 1.6	Chuanxiong rhizoma	30.7 ± 3.2
Mulberry leaf	65.6 ± 1.2	Cinnamomi cortex	27.0 ± 2.4
Anemarrhenae rhizoma	64.4 ± 1.6	Polygoni multiflori radix praeparata	26.3 ± 1.9
Polygoni cuspidati rhizoma et radix	50.3 ± 1.1	Salviae miltiorrhizae radix et rhizoma	25.3 ± 0.6
Puerariae lobatae radix	44.5 ± 1.7	Astragali radix	24.6 ± 1.59
Angelicae sinensis radix	37.0 ± 3.6	—	—

**Table 3:** Docking results of six small-molecule compounds with lipase.

Compounds	Binding energy (Kcal/mol)	Hydrogen-bonds	Other amino acid residues
(−)-Epigallocatechin gallate	−7.43	SER128, LYS132, ASN131, and LEU93	PRO134, PRO67, LEU133, ASP160, LYS66, TYR95, and GLY94
(−)-Epigallocatechin	−6.26	SER128, LYS132, LYS66, and LEU275	LEU133, PRO134, TYR95, PRO67, ARG276, ASN131, and SAP160
(−)-Epicatechin gallate	−7.89	SER128, LYS132, ASN131, and LYS66	PRO67, TYR95, LEU133, ASP160, and PRO134
Epicatechin	−6.48	SER128, PRO67, and ASP160	LYS66, LYS132, LEU133, PRO134, TYR95, ARG161, and ASN131
Rosmarinic acid	−6.19	ARG272 and LYS132	SER273, LEU275, ARG276, TYR95, PRO67, LEU133, SER128, ASN131, LEU93, LYS66, and PRO134
(+)-Catechin	−6.30	LEU275, LEU93, and ASP160	TYR95, GLY94, LYS66, ARG276, ARG161, ASN131, SER128, LYS132, LEU133, PRO67, and PRO134

## Data Availability

All data generated or analysed during this study are included in this article.
